The article "The Innovative Use of Ureter Catheter in the Surgery of Obstructive Uropathy" was published in 2021. Journal: Comput Math Methods Med.

# The Innovative Use of Ureter Catheter in the Surgery of Obstructive Uropathy

**DOI:** 10.1155/2021/6668415

**Published:** 2021-03-17

**Authors:** Xiangcheng Zhan, Ding Liu, Guangchun Wang, Haimin Zhang, Aimaitiaji Kadier, Xudong Yao, Yunfei Xu

**Affiliations:** Department of Urology, Shanghai Tenth People's Hospital, Tongji University School of Medicine, Shanghai 200072, China

## Abstract

**Purpose:**

Relieving obstruction and protecting renal function are the main therapeutic purposes of obstructive uropathy which often involve surgical treatment, and the ureter catheter is one of the surgical instruments commonly used in surgery. We aimed to explore the innovative use of a ureter catheter in the surgery of obstructive uropathy.

**Methods:**

We used a ureteral catheter to innovate the surgical procedure of the most common causes of obstructive uropathy: ureteral calculi and stricture, establishing an internal circulation system (ICS), proposing a three-step dilatation method, and reviewing their effects on patients. Furthermore, we introduced a simple real-time intrapelvic pressure measurement device to monitor intrarenal pressure during operation.

**Results:**

Postoperative laboratory examination showed that blood CRP, leukocyte neutrophil level, changes in the hemoglobin, urine occult blood, and positive rate of urine culture in the ICS group are significantly lower than those in the control group, corresponding to a lower incidence of bleeding and infection-related complications clinically. A three-month follow-up revealed 1/3 rate of ureteral stricture in the ICS group comparing to the control. We applied the three-step dilatation in patients with severe stenosis in which the balloon could not pass; the overall effective rate was 90.9%. The pressure of the renal pelvis was displayed on the monitor in real time. The surgeon could estimate the degree of filling of the renal pelvis and adjust the intake volume through the data.

**Conclusion:**

The innovative application of ureteral catheters in the operation of obstructive uropathy can realize the real-time monitor of intraoperative renal pelvis pressure, reduce the incidence of lithotripsy postoperative complications, and expand the indications of balloon dilatation in ureteral stricture, which has certain clinical significance.

## 1. Introduction

Obstructive uropathy, characterized by prevention of urine flow, refers to urinary tract obstruction caused by various reasons (such as lithiasis, infections, and tumors) which may lead to a series of pathophysiological changes and clinical symptoms. Among them, acute diseases include acute kidney injury (AKI), urosepsis which are life threatening, and long-term urinary flow obstruction which will cause different degrees of decline in renal function [1]. Relieving obstruction and protecting renal function are the main therapeutic purposes of obstructive uropathy which often involve surgical treatment, and the ureter catheter is one of the surgical instruments commonly used in surgery.

The article "The Innovative Use of Ureter Catheter in the Surgery of Obstructive Uropathy" was published in 2021. Journal: Comput Math Methods Med.

In 1967, the use of a 19-month-long indwelling ureteral silicone tube was first described by urologist Zimskind et al. [2], representing the prelude to the official clinical application of a ureteral catheter. The ureteral catheter is a passive dilated tube that facilitates the drainage of urine from the ureter and ureteral orifice into the bladder. It is commonly used in urologic practice including (1) to relieve ureteral obstruction caused by stone, cancer, and deformity; (2) the treatment of ureter leak or anastomosis; and (3) revealing the shape of a renal assembly system by reverse injection of water. The original ureteral catheter is made of polyethylene materials with a straight shape; the upper end stays in the renal pelvis and the lower end extends outside the urethra. But the straight-shape design made it prone to displacement; to solve this problem, Finney described a ureteral catheter fitted with a curl on both sides which is known as a double pigtail stent or “double-J” ureteral catheter [3].

Ureteral catheters underwent over half a century of development and improvement on their designs, materials, and coating for better comfort and fewer complications; the original straight-shaped design was gradually replaced. However, in our clinical practice, we found that the straight-shaped ureteral catheter can serve as a unique auxiliary surgical instrument in the treatment of obstructive uropathy.

## 2. Methods

### 2.1. Application of Ureteral Catheter in Surgery of Urolithiasis

In our clinical practice, we established an internal circulation system (ICS) by preinserting a 5 Fr ureteral catheter. Before the insert, ureteroscopy is performed (with 8/9.8 Fr Wolf ureteroscope) combined with CT scan to assess stone obstruction and ureteral condition. Then, we retreat the ureteroscope to the ureteral orifice and place a 5 Fr ureteral catheter. We reenter the ureter to make sure the catheter neither slips nor touches the stone. Then, we operate the rigid ureteroscope to the obstruction level and adjust the position of the stent under the surgical field of vision to prevent the damage by the laser. The intake valve is opened constantly to ensure the water drainage of the stent is smooth; internal circulation system is successfully established. Holmium laser lithotripsy is performed until the stone is fragmented below 1 mm in diameter.

The article "The Innovative Use of Ureter Catheter in the Surgery of Obstructive Uropathy" was published in 2021. Journal: Comput Math Methods Med.

We developed ICS and applied it to the clinic in 2019 and successfully completed 50 cases of obstructive ureteral calculi surgery under the ICS system. We selected 50 patients undergoing obstructive ureteral calculus surgery as the control group to compare the operation time and postoperative indexes which reveals the occurrence of complications such as postoperative infection and bleeding. All 100 operations were performed by the same surgeon.

### 2.2. Three-Step Dilatation in Treatment with Ureteral Stricture

(Step 1) *Cold cutting of ureteral catheter*: trim the end of the ureteral catheter with a scalpel to give it a sharp angle of 30° (Figure 1). Then, deliver the stent to the stricture along the guide wire under the ureteroscope and cut the narrow ring with the sharp end. The trimmed stricture is triangular.
(Step 2) *Ureteroscopic dilatation*: operate the ureteroscope gently through the triangular wound to dilate the stricture with the scope.
(Step 3) *Balloon dilatation*: use the dilate balloon to dilate the stricture 1-2 times with the pressure less than 25 kPa for 5 minutes. Two double-J ureteral catheters are placed after the dilatation.

### 2.3. Construction of Simple Real-Time Intrapelvic Pressure Measuring Device

For patients undergoing percutaneous nephrolithotripsy, we perform a percutaneous renal pelvic puncture and place a 5 Fr ureteral catheter. The distal end is connected to a 0.9% saline bag. Another ureteral catheter is placed in the renal pelvis under the ureteroscope, and the distal end of the catheter is connected to the pressure transducer (DPT-248 Utah Medical Products, USA) and the monitor. When the saline bag is lifted to different heights, the pressure value on the monitor corresponds to the pressure in the renal pelvis of different cmH_2_O. As the upper catheter is replaced with the percutaneous nephroscope to perform lithotripsy, the retrograde-placed ureteral catheter stays in the renal pelvis, and real-time renal pressure data is displayed on the screen for intraoperative monitoring (Figure 2).

## 3. Results

### 3.1. Effect of Internal Circulation System on Surgery

We can see from the figure, compared with the traditional single-channel operation, that the surgical field of view under the ICS was clearer, with less fragments and bubbles. Moreover, the relationship between the stone, the ureteral wall, and the laser fiber is more distinct, which helped the urologist avoid perforation and significantly shortened the fragmentation time (Figure 3).

### 3.2. Effect of Internal Circulation System on Patients

Blood and urine samples were collected the day after surgery. Blood test showed lower CRP, leukocyte, and neutrophil level in patients undergoing surgery under ICS than the patients in the control group. In the meantime, urine routine and culture also revealed that the incidence of urinary tract infection (UTI) in the control group (22%) is 2.2 times that of the ICS group (10%), which indicates that performing ureteroscopic lithotripsy under ICS can effectively reduce the incidence of postoperative infection.

The article "The Innovative Use of Ureter Catheter in the Surgery of Obstructive Uropathy" was published in 2021. Journal: Comput Math Methods Med.

Bleeding is another surgical complication of our concern. Since the ureteroscopic lithotripsy bleeding is mainly due to urethral injury, we compared results of blood hemoglobin changes and urine occult blood (BLD) level of the two groups. Patients in the ICS group had a higher HB level and lower BLD level than those in the control group, indicating less urethral injury and bleeding in the ICS group (Figure 4).

These patients were also followed up three months after surgery with a urinary ultrasound and a nephrogram. For patients with hydronephrosis and a marked decline in kidney function, ureteroscopy was performed to find out whether there was ureteral stricture. It turned out that 6 patients in the control group and 2 in the ICS group are diagnosed with ureteral stricture.

### 3.3. Clinical Application of Three-Step Dilatation

In this study, we used a three-step dilatation in 11 patients with ureteral stricture, including 9 males and 2 females, with an average age of 52.5 years. Surgical effects were divided into cure, improvement, and ineffective, according to clinical criteria. As a result, 4 patients were cured by this method, 6 were improved, and the remaining 1 was ineffective, and thus, the overall effective rate was 90.9%. In 7 patients with positive effects, 6 had upper segment stenosis and 1 in the lower segment; 3 of them found polyps in the ureter. To the extent of hydronephrosis, 1 case was mild, 2 cases were moderate, and 4 cases were severe. Of the 4 ineffective patients, three were accompanied by severe hydronephrosis and the formation of inflammatory polyps in the ureter, and the remaining case only had mild hydronephrosis (Table 1). For reasons of endoscopic operation, we cannot measure the exact length of the stricture segment.

### 3.4. Clinical Application of Real-Time Intrapelvic Pressure Measuring Device

We applied the real-time intrarenal pelvis pressure measuring device in percutaneous nephroscopy. The pressure of the renal pelvis was displayed on the monitor in real time. The surgeon could estimate the degree of filling of the renal pelvis and adjust the intake volume through the data.

## 4. Discussion

As a urologist, how to apply our surgical instruments wisely is an indispensable quality in the treatment of urological diseases. A ureter stent is one of the most commonly used instruments to brace the ureter and ensure urine flow. In this study, we mainly introduce our application experience in the surgery of obstructive uropathy.

The article "The Innovative Use of Ureter Catheter in the Surgery of Obstructive Uropathy" was published in 2021. Journal: Comput Math Methods Med.

Urinary calculus is the main cause of urinary obstruction in adults as well as what we commonly encounter in urology surgery, and its incidence has been increased worldwide [4, 5]. Nowadays, ureteroscopy is proven to be a powerful weapon in the treatment of ureter calculi. Meanwhile, a series of complications caused by ureteroscopy have received increased attention including early postoperative hematuria, urosepsis, and urinary tract injury, along with late postoperative ureteral stricture, hydronephrosis, and kidney function decline, etc. [6–10]. In addition to the stone itself, there are also iatrogenic causes in the occurrence of complications, such as nuclear surgical field of vision, prolonged operation time, and applying energy on the mucosa. In practice, we find that using a ureteral catheter may be an effective way to solve the problems above.

The incarceration of the stone often causes local edema in the ureter [11]. When the ureteroscope is inserted, a confined space is formed between the scope and the stone. Therefore, when carrying out subsequent lithotripsy, the stone fragments will blur the vision of the operation which makes the boundary between the stone and the ureteral wall unclear so that the mucous is easily damaged. If the water valve is opened for flushing, it may cause the local or intrarenal pressure to rise sharply. In addition, continued use of lasers increases local water temperature which may cause thermal damage to the ureter wall which increases the risk of postoperative ureteral stricture [12]. Hence, we came up with the idea of placing a 5 Fr ureter stent. Firstly, the small debris during the lithotripsy is excreted through the stent, maintaining a clear surgical vision and thus reducing the damage to the ureteral mucosa. Secondly, the ICS enables the surgeon to rinse continuously, and smooth drainage reduces local pressure and the heat generated by the laser which increase the efficiency of lithotripsy while minimizing the probability of thermal damage.

The results of laboratory examination after the surgery reflect the occurrence of early postoperative complications. Our primary concern is postoperative infection and bleeding. UTI after ureteroscopy is not rare. According to a global study of 11,885 patients who underwent ureteroscopy by the clinical research office of the Endourological Society (CROES), the incidence of postoperative UTI is 1% [13], and the severe cases can progress to urosepsis which endangers patients' lives. Ureteral calculi are the cause of infection itself while longer operative time is one of the risk factors as well [14]. In fact, we find that the mean lithotripsy time in the control group is 23.7 minutes while only 16.6 minutes in the ICS group, which reveals that the use of ICS significantly reduces the lithotripsy time by 30%. The results of urine routine and urine culture were used to monitor the occurrence of UTI, and the incidence of UTI is lower in the ICS group. Furthermore, blood test results also showed infection indexes such as CRP and the blood leukocyte level as significantly lower in the ICS group than in the control group, suggesting that ICS can effectively reduce the risk of postoperative infection. Previous studies reported that bleeding happens in about 1%-2.5% cases caused by ureter injuries with various injuries [6, 13, 15]. We observed fewer ureteral injuries and bleeding in the ICS group during the operation. A postoperative BLD test showed that the degree of hematuria in the ICS group was significantly lower than that in the control group. At the same time, the blood test showed that hemoglobin decline is lower in the ICS group as well, suggesting that the use of ICS can reduce bleeding risk and blood loss of the patient. In the study of late postoperative complications, the ICS group also showed less ureteral stricture during the three-month follow-up and review.

The article "The Innovative Use of Ureter Catheter in the Surgery of Obstructive Uropathy" was published in 2021. Journal: Comput Math Methods Med.

Overall, ICS provided a clearer surgical field and extra water loop which enable the surgeon to shorten the operating time and reduce the incidence of bleeding, infection, and ureteral stricture. However, the establishment of ICS has certain requirements for ureteral conditions. For patients with ureteral difficulties, forcibly placing a ureteral catheter tube may increase the risk of ureteral perforation and even avulsion. Therefore, it is important to perform ureteroscopy to understand the condition of the ureter. This depends on the experience and judgment of the surgeon. The incidence of complications in our clinical data was also above average; this could be attributed to our criteria for patient selection.

Congenital factors and secondary causes, such as surgical injuries, stones, infections, and trauma, can cause benign ureteral stricture [16]. Balloon dilatation is considered to be the most suitable method for the endoscopic treatment of ureteral stricture due to its fewer complications and low cost [17] with a high technical success rate up to 89% [18]. But sometimes, we will encounter the situation where the stricture segment is so narrow that it can only allow the guide wire to pass and the balloon cannot be inserted. At this time, surgeons often choose alternative surgical procedures such as endoureterotomy and open surgery which bring more trauma, complications, and costs to patients. Herein, we innovatively use ureter stents to help surgeons out of this dilemma. Our innovative three-step approach is aimed at dilatating the stricture segment gradually and gently to eventually get the balloon through. The hollow design of the ureteral catheter allows it to move in the direction of the guide wire, avoiding the perforation and the formation of the false passage in the ureter. Trimming the distal end of the stent to a 30-degree angle, the narrow ring is cut by a puncture at multiple angles which plays a similar role of a cold knife incision. After the second step of dilatation and confirmation of the correct channel, the subsequent procedure is the same as conventional balloon dilatation. Regardless of traditional open surgery or endoureterotomy, the surgical instruments (such as a cold knife and laser) and the surgeon's surgical experience are highly demanded. Our three-step dilatation takes advantage of the characteristics of the ureteral catheter and expands the indication of the balloon dilatation. In fact, clinical application results showed encouraging effects; the overall improvement rate exceeded 90%, proving that the three-step dilatation is a feasible and innovative improvement for traditional balloon dilatation.

The article "The Innovative Use of Ureter Catheter in the Surgery of Obstructive Uropathy" was published in 2021. Journal: Comput Math Methods Med.

Prolonged upper urinary tract obstruction and surgical irrigation will lead to increased pressure of the renal pelvis. When the intrapelvic pressure exceeds 40 cm H_2_O, the contents of the renal pelvis system go beyond its limit, initiating pyelosinus, pyelovenous, pyelolymphatic backflow, and/or irrigation fluid absorption [19–21]. Increased intrapelvic pressure has been proven to be a major risk factor for postoperative fever and urosepsis [22]. Moreover, excessive fluid absorption leads to fluid overload, hyponatremia, and cardiovascular instability [23]. Actually, backflow and fluid absorption are not uncommon in renal and ureteral surgeries; Malhotra et al. reported that fluid absorption occurred in 78% percutaneous nephrolithotripsy cases with the mean volume of 696.7 ml [21]. Based on our understanding of the importance of intraoperative renal pelvis pressure, we constructed this simple real-time pressure measuring device. The ureteral catheter is widely used in percutaneous nephrolithotripsy to fill the renal pelvis during percutaneous puncture and prevent gravel from falling into the ureter. The use of a ureteral catheter tube to construct a pressure measurement device saves the need for additional surgical instruments and facilitates real-time intraoperative pressure measurement. Actually, in our application, we found individual differences in the pressure produced by the same height of water column on the renal pelvis, which is possibly related to differences in anatomical structure and partial flow back to the bladder through the gap between the ureter and the stent. Therefore, the pressure measured by our device is not as accurate as the classical pressure measurement methods, such as the Whitaker test. The Whitaker test reflects the relative pressure in the renal pelvis by measuring the pressure difference between the renal pelvis and the bladder under the condition of constant flow perfusion, which is also used for the etiological diagnosis of upper urinary tract obstruction [24]. Compared with the traditional renal pelvis pressure measurement and diagnosis methods represented by the Whitaker test, the main purpose of the pressure measurement device we built is to provide effective reflection of pelvis pressure during surgery rather than a well-defined diagnosis, helping the surgeon control the intraoperative pressure, thereby reducing the incidence of intraoperative and postoperative complications. As an invasive operation, the real-time intrapelvic pressure measuring device is currently only used in patients with upper urinary calculi carrying renal fistula or during percutaneous nephrolithotripsy procedure.

The article "The Innovative Use of Ureter Catheter in the Surgery of Obstructive Uropathy" was published in 2021. Journal: Comput Math Methods Med.

## 5. Conclusion

The purpose of the current study was to purpose the innovative use of a ureteral catheter during our surgical practice of obstructive uropathy and explore its clinical value for patients. We constructed the internal circulation system and simple real-time intrapelvic pressure measuring device in the surgery of urinary stone disease which enabled the surgeon to monitor the intrarenal pressure during surgery, shortened operation time, lowered postoperative bleeding, and infection-related indexes and let patients benefit from fewer complications. The three-step dilatation characterized by using a trimmed ureteral catheter as a cold knife expanded the indication of balloon dilatation without affecting its effective rate. Taken together, our study suggests that the innovative use of the ureteral catheter has important clinical application value and promotion value in the surgery of obstructive uropathy.

## Figures and Tables

**Figure 1:** Using a ureter as a cold knife in ureter dilatation. We trimmed the distal end of the ureter catheter to give it an angle of 30°, which can be used as a cold knife to realize the first-step dilatation.

**Figure 2:** Construction of simple real-time intrapelvic pressure measuring device. (a) When the percutaneous pelvic tunnel is formed, we placed a 5 Fr ureteral catheter which is connected to a 0.9% saline bag before the fragmentation. Pelvic pressure at different heights can be revealed on the monitor through the pressure transducer. (b) Real-time intrapelvic pressure data is displayed on the screen during the fragmentation to enable the surgeon monitor the intrapelvic pressure.

The article "The Innovative Use of Ureter Catheter in the Surgery of Obstructive Uropathy" was published in 2021. Journal: Comput Math Methods Med.

**Figure 3:** Clinical application of ICS. We collected intraoperative images of patients operated under ICS. (a) shows that the surgical view was blurred due to insufficient circulation. When the ureteral catheter was inserted, water drainage was fluent with extra tunnel (b), and surgical view became clearer because of the constant water circulation (c). (d) The fragmentation time is significantly shortened in patients with ICS. Mean ± SEM, *n* = 50; ^∗∗∗∗^*P* < 0.0001 designates significant difference when compared to the control.

**Figure 4:** Postoperative blood indexes. All patients received blood and urinary test one day after the surgery. The outcome showed that blood CRP, blood leukocyte, neutrophil, PLT, reduction of HB, and BLD of the ICS group are significantly lower than those of the control group. Mean ± SEM, *n* = 50; ^∗^*P* < 0.05, ^∗∗^*P* < 0.01, and ^∗∗∗∗^*P* < 0.0001 designate significant differences when compared to the control.

**Table 1:** Clinical data of three-step dilatation.

	Cure	Improve	Ineffective
Number	4	6	1
Average age	52.75	52	55
Sex (male/female)	3/1	5/1	1/0
Location (upper/lower)	4/0	4/2	0/1
Cases with polyps	1	2	1
Hydronephrosis degree (mild/moderate/severe)	2/2/0	0/2/4	0/0/1

## Data Availability

The data could be provided when any other researchers need it.
